RETRACTED

# The impact of different weed management strategies on weed flora of wheat-based cropping systems

**DOI:** 10.1371/journal.pone.0247137

**Published:** 2021-02-18

**Authors:** Muhammad Shahzad, Khawar Jabran, Mubshar Hussain, Muhammad Aown Sammar Raza, Leonard Wijaya, Mohamed A. El-Sheikh, Mohammed Nasser Alyemeni

**Affiliations:** 1 Department of Agronomy, Bahauddin Zakariya University, Multan, Pakistan; 2 Department of Agronomy, University College of Agriculture & Environmental Sciences, The Islamia University of Bahawalpur, Bahawalpur, Pakistan; 3 Department of Plant Protection, Niğde Ömer Halisdemir University, Niğde, Turkey; 4 Department of Botany and Microbiology, College of Science, King Saud University, Riyadh, Saudi Arabia; Harran University, TURKEY

## Abstract

The world population will rise in future, which would demand more wheat production to fulfil dietary needs of wheat-dependent population of the world. Food security in wheat-dependent regions will greatly rely on wheat productivity. Weed infestation is a major constraint reducing wheat productivity globally. Nonetheless, cropping systems and weed management strategies strongly influence weed infestation in modern agriculture. Herbicides are the key weed management tool in conventional agriculture. However, frequent use of herbicides have resulted in the evolution of herbicide-resistance weeds, which made weed management a challenging task. Sustainable and eco-friendly weed management strategies shift weed-crop competition in the favour of crop plants. Limited studies have evaluated the interactive effect of cropping systems and weed management strategies on weed flora of wheat-based cropping systems (WBCSs). This two-year study evaluated the impact of different weed management strategies (WMSs) on weed flora of WBCSs, i.e., fallow-wheat (FW), rice-wheat (RW), cotton-wheat (CW), mungbean-wheat (MW) and sorghum-wheat (SW). The WMSs included in the study were, false seedbed, allelopathic water extracts and herbicide application, while weed-free and weedy-check were maintained as control treatments. Data relating to diversity and density of individual and total broadleaved and narrow-leaved weeds were recorded. The WBCSs, WMSs and their interaction significantly altered diversity and density of individual, total, broadleaved and narrow-leaved weeds. Weed-free and weedy-check treatments recorded the lowest and the highest values of diversity and density of individual, total, broadleaved and narrow-leaved weeds. Herbicide application effectively reduced density and diversity of weeds. Allelopathic water extracts and false seedbed proved less effective than herbicides. On the other hand, SW cropping system not only reduced weed density but also limited the weed flora. It is concluded that false seedbed and SW cropping system can be efficiently used to manage weeds in WBCSs. However, long-term studies are needed to infer the impact of SW cropping system and false seedbed on soil properties, soil microbes and productivity of wheat crop.

RETRACTED

## Introduction

Wheat (*Triticum aestivum* L.) is the most widely cultivated cereal around the world with annual cultivation on 220.41 million hectares and production of 734 million tons [1]. Wheat feeds over one-fifth global population by serving as staple food [2, 3]. It provides ~19% of daily caloric intakes and 21% of the dietary protein globally [4]. Wheat production will significantly influence global food security than any other crop due to its high popularity, and widespread production and consumption [1, 2, 5]. It is estimated that if world population grows with the present day rate, it will add 2.4 billion human on earth until 2050 [6]. Increasing population in wheat-dependent regions would demand more wheat production [5]. Wheat production must be increased by 1.7% annually to feed the massive population of globe during 2050 [7]. However, global annual expansion in wheat production is 1.1% [8]. Nonetheless, wheat production is becoming stagnant in several regions of the world [9]. Delayed harvesting of kharif crops [10], use of old varieties [10], improper seed rate and row spacing [11–15], poor fertilizer use efficiency [16], weed infestation [17] and drought stress [18, 19] are regarded as the main reasons of stagnant wheat yields.

Generally, wheat is part of different cropping systems in various regions of the world [17, 20]. Rice-wheat and cotton-wheat cropping systems share 60% of cultivated wheat area globally [21]. Weeds are among the major reasons decreasing crop productivity in wheat-based cropping systems. Weeds offer significant hurdles in sustainable agricultural production [17, 22–24]. Weeds interfere with crop production practices and incur significant yield and quality losses [17, 22, 25, 26]. Several agronomic practices are required to create favourable environment for different crops in modern agricultural systems; however, these activities favour weed proliferation [17, 27, 28]. Soil types and cultivation systems along with agronomic practices strongly influence weed flora in different cropping systems [17, 27, 28].

Continuous growing of same crop in a cropping system results in the prevalence of the best-suited weeds [17, 29]. Nonetheless, various cropping systems results in the prevalence of specific weeds due to opted agronomic practices [17]. For instance, fallow-wheat and mungbean-wheat cropping systems favour grassy and broadleaved weeds, respectively [17]. Moreover, sorghum-wheat cropping system favoured fat hen, whereas common goosefoot, broadleaved dock and salt marsh were favoured by rice-wheat cropping system. Likewise, broad-leaved dock, salt marsh, yellow sweet clover, rabbit foot grass, perennial sow thistle, corn spurry and bermuda grass were favoured by fallow-wheat cropping system [17]. Similarly, it has been reported that rice-wheat cropping system favoured grassy weeds and suppressed broadleaved weeds [30]. These best-adapted weed species in such cropping systems are difficult to manage by existing weed management practices due to herbicide resistance, labour costs and environmental pollution.

RETRACTED

Manual weed control is regarded as the best and sustainable weed management option; however, increasing costs and labour shortage have rendered this technique ineffective [31]. Hiking costs of manual weed control have forced farmers to adopt alternative weed management strategies. Weed management with herbicides is an easiest and most successful method [32]. Herbicides have played a significant role in modern agriculture for weed management [33]. Excessive use of herbicides have resulted in the rapid evolution of herbicide-resistant weeds [34–36]. Globally, 512 herbicide resistant weed biotypes have been recorded till date [37]. Excessive use of herbicides have evolved resistant weeds, which are difficult to manage with the available herbicides [34–36]. A recent study has called to integrate conventional weed management practices, molecular biology and new weed management approaches to manage herbicide resistance [38].

The primary principle of sustainable weed management strategies should be decreasing or altering the weed-crop competition in favour of crop plants [17, 39, 40]. Therefore, crop rotation, allelopathy and false seedbed preparation may be exploited as weed management strategies. These methods can seize weed sprouting and reproduction resulting in decreased weed-crop competition [41–44]. Crop rotation could lower weed pressure; however, thorough understanding of weed flora is needed to include crops in rotation for weed management [17, 45]. False seedbed preparation could control annual weeds persisting in different cropping systems [46]. False seedbed lowers weed density before crop sowing; thus, can be successfully used to lower weed-crop competition [44, 46].

Allelopathy is another important weed management technique, which is eco-friendly and successfully used in different crops. Weeds are controlled by using allelopathic mulches, crop rotation, intercropping and foliar application of allelopathic crop water extracts [42, 43, 47, 48]. Sorghum, eucalyptus, mulberry, and sunflower are some of the allelopathic crops whose weed control potential has been described in literature [17, 42, 48–52]. Different allelochmeicals are present in sorghum (phenolics, and sorgoleone), sunflower (terpenes and phenolic compounds) and mulberry (steroids, phenols and tannins), which enable them to control weeds with differential success [50, 53–55]. It has been proved that sorghum metabolites effectively control broadleaf weeds than grasses [56].

RETRACTED

It is evident from the above discussion that weed management practices should be revised based on existing weed flora in agricultural fields rather than relying on existing options. This study investigated the impacts of different weed management strategies on weed flora of various wheat-based cropping systems. It was hypothesized that cropping systems and weed management strategies will significantly differ for weed flora. The results will help in the weed management and selection of the most suitable wheat-based cropping system with less weed pressure.

## Materials and methods

### Experimental location description

Experimental site is located at 30.2°N latitude, 71.43°E longitude and at an altitude of 122 m above mean sea level in Bahauddin Zakariya University, Multan, Pakistan. The soil of the experimental site was silty-clay and slightly saline in nature. The chemical analysis revealed that organic matter contents were 0.54 and 0.59%, pH was 8.35 and 8.42, and EC was 3.29 and 3.31 dS m^−1^ during 1^st^ and 2^nd^ year, respectively. Total available nitrogen was 0.03 and 0.04 mg/l, total available phosphorus was 8.75 and 8.87 mg/l and total available potassium was 180 and 195 mg/l during 1^st^ and 2^nd^ year, respectively. The weather data of the experimental site for both years is presented in Fig 1. No field permit was necessary to conduct the study and there were no endangered species involved in the experiments.

**Fig 1:** Weather data of the experimental site during both experimental years.

### Treatments, layout, and experimental details

The experiment consisted of five wheat-based cropping systems (WBCSs) and three weed management strategies (WMSs) along with two controls for comparison of WMSs. The WBCSs were fallow-wheat (FW), rice-wheat (RW), cotton-wheat (CW), mungbean-wheat (MW) and sorghum-wheat (SW). The WMSs were false seedbed, allelopathic plant water extracts, herbicide application, whereas controls were weedy-check (no weed control) and weed-free (100% weed control). The experiment was laid out according to randomized complete block design (split-plot arrangements) with three replications. The WBCSs were kept in main-plots and WMSs were randomized in sub-plots. Each plot had an area of 15 m^2^. No crop, rice, cotton mungbean and sorghum were sown during summer season in FW, RW, CW, MW and SW cropping systems, respectively, which were followed by wheat in winter season. Weeds were manually eradicated in weed-free treatment, while no weeding was done in weedy-check treatment throughout the growing season. In case of stale/false seedbed, seedbed was prepared as a routine seedbed but kept fallow for seven days, after that field was ploughed again and wheat was sown. Bromoxynil + MCPA (Bromox 40EC) (200 g/L bromoxynil present as octanoate 200 g/L MCPA present as ethyl hexyl ester solvent 343 g/L liquid hydrocarbon) was applied at recommended dose (1.25 L ha^-1^: 500 g a.i. ha^-1^) in herbicide application treatment. Herbicide was applied after 1^st^ irrigation, i.e., when wheat reached to four leaf stage. In allelopathic water extracts, sorghum, mulberry, sunflower and eucalyptus water extracts were mixed in equal quantities and applied at the suggested dose (12 L ha^-1^) at four leaf stage of wheat crop. The herbicide and allelopathic water extracts were applied in the direction of wind by using Knapsack hand sprayer fitted with T-jet nozzle.

RETRACTED

### Crop husbandry

In each growing season, pre-soaking irrigation of 10 cm was applied to the experimental field prior to seedbed preparation. Seed rates for wheat, cotton, rice (nursery), mungbean and sorghum were kept 125 kg ha^-1^, 25 kg ha^-1^, 40 g m^-2^, 20 kg ha^-1^ and 10 kg ha^-1^, respectively. The production technology adopted for all these crops were same as described in Shahzad et al. [17, 40]. All crops were harvested at their physiological maturity.

### Procedures to record data

Weeds diversity was measured by visiting the experimental field throughout growing period of wheat crop and densities of individual weeds were recorded at 60 days after sowing. Weed diversity was recorded by observing all species in 1 m^2^ at three random places in each experimental unit and averaged. To measure the densities of total, broadleaved, grassy and individual weeds, the method adopted by Onen et al. [57] was followed. Briefly, a 0.5 × 0.5 m quadrate was randomly placed at three different places in each experimental unit. Total number of weeds were recorded, averaged and converted to plants m^-2^ by unitary method. The observed weed species for density were separated into their individual classes to record the density of broadleaved, grassy and individual weeds.

### Statistical analysis

Data recorded on total, broadleaved, grassy and individual weed diversity were analysed using statistical software *STATISTIX 8*.*1*. The data were tested for normality first by Shapiro-Wilk normality test and non-normal variables were normalized by Arcsine transformation. Differences among years were tested by paired *t* test, which was significant. Therefore, data of both years were analysed, presented and interpreted, separately. Two-way analysis of variance (ANOVA) was used to test the significance in the data [58]. Least significant difference post-hoc test was used to separate means where ANOVA indicated significant differences. Moreover, Microsoft Excel program 2016 was used to plot the graphs for graphical presentation of the data.

RETRACTED

## Results

### Diversity and density of total weeds

Weed diversity was significantly affected by different WBCSs and WMSs (Fig 2). The highest weed diversity was recorded for RW system, whereas CW observed the lowest weed diversity during both years. Similarly, the highest and the lowest weed diversity was recorded for weedy-check and herbicide application treatments, respectively (Fig 2).

**Fig 2:** Effect of different weed management strategies on weed diversity (number of weed species) under different wheat based cropping systems during (a) 2012–2013 and (b) 2013–2014 ± S.E.

Herbicide application in MW cropping system during 1^st^ year and SW cropping system during 2^nd^ year recorded the lowest weed diversity. Similarly, RW cropping system with weedy-check and false seedbed during 1^st^ year and RW cropping system with false seedbed had the highest weed diversity during 2^nd^ year of the study (Fig 2).

The WMSs significantly reduced total weeds density compared with weedy-check. The highest (>95%) reduction in total weeds’ density was recorded for herbicide application, which was followed by false seedbed. However, allelopathic extracts resulted in lower reduction of total weeds’ density compared with weedy-check during both years (Table 1).

**Table 1:** Effect of different weed management strategies on total weeds, broadleaved and narrow-leaved weeds’ density (m^-2^) under different wheat-based cropping systems during 2012–2013 and 2013–2014.

Cropping systems	2012–2013					Means	2013–2014					Means
	WF	WC	FS	CC	AWE		WF	WC	FS	CC	AWE	
	Total Weeds											
**FW**	-	185.67 a	44.67 f	3.33 j	88.33 d	**64.40 a**	**-**	103.33b	40.33 f	6.33 kl	35.67 g	**37.13 b**
**RW**	-	184.00 a	46.00 f	4.33 j	73.00 e	**61.47 b**	**-**	168.00a	56.00 d	12.00 j	65.33 c	**60.27 a**
**CW**	-	115.00 c	25.00 h	3.00 j	29.00 h	**34.40 d**	**-**	48.00 e	19.00 i	5.00 lm	19.33 i	**18.27 d**
**MW**	-	146.33 b	37.33 g	2.33 j	47.67 f	**46.73 c**	**-**	67.00 c	16.00 i	4.33 lm	19.00 i	**21.27 c**
**SW**	-	69.33 e	17.00 i	2.00 j	25.33 h	**22.73 e**	**-**	24.33 h	11.67 j	2.00 mn	8.67 jk	**9.33 e**
**Means**	**-**	**140.07 a**	**34.00 c**	**3.00 d**	**52.67 b**		**-**	**82.13 a**	**28.60 b**	**5.93 c**	**29.60 b**	
			**(69.22)**	**(97.28)**	**(52.32)**				**(65.17)**	**(92.79)**	**(63.95)**	
**LSD 5%**	**W = 2.12, C = 2.12, W×C = 4.75**						**W = 1.49, C = 1.49, W×C = 3.34**					
	**Broad leaved weeds**											
**FW**	**-**	164.00 a	36.00 h	**-**	83.00 e	**56.60a**	**-**	83.67 b	30.67 f	**-**	26.00 g	**28.07 b**
**RW**	**-**	151.00 b	34.33 h	**-**	60.33 f	**49.13b**	**-**	136.33a	35.67 e	1.00 m	45.33 d	**43.67 a**
**CW**	**-**	101.00 d	21.00 i	**-**	22.67 i	**28.93d**	**-**	37.67 e	15.00 i	**-**	9.67 jk	**12.47 d**
**MW**	**-**	127.00 c	32.33 h	**-**	41.00 g	**40.07c**	**-**	57.67 c	11.67 j	**-**	16.33 i	**17.13 c**
**SW**	**-**	62.33 f	14.00 j	**-**	21.67 i	**19.60e**	**-**	20.00 h	9.00 kl	**-**	6.67 l	**7.13 e**
**Means**	**-**	**121.07 a**	**27.53 c**	**-**	**45.73 b**		**-**	**67.07 a**	**20.40 b**	**0.20 c**	**20.80 b**	
			**(77.37)**	**(100)**	**(62.22)**				**(69.58)**	**(99.70)**	**(68.98)**	
**LSD 5%**	**W = 1.87, C = 1.87, W×C = 4.17**						**W = 1.08, C = 1.08, W×C = 2.42**					
	**Narrow leaved weeds**											
**FW**	-	21.67 b	8.67 f	3.33 l-n	5.33 h-j	**7.80 b**	**-**	19.67 b	9.67 c	6.33 d	9.67 c	**9.07 b**
**RW**	-	33.00 a	11.67 e	4.33 j-l	12.67 de	**12.33a**	**-**	31.67 a	20.33 b	11.00 c	20.00 b	**16.60 a**
**CW**	-	14.00 d	4.00 j-l	3.00 l-n	6.33 g-i	**5.47 d**	**-**	10.33 c	4.00 e-g	5.00 de	9.67 c	**5.80 c**
**MW**	-	19.33 c	5.00 i-k	2.33 mn	6.67 gh	**6.67 c**	**-**	9.33 c	4.33 d-f	4.33 d-f	2.67 fg	**4.13 d**
**SW**	-	7.00 g	3.00 l-n	2.00 n	3.67 k-m	**3.13 e**	**-**	4.33 d-f	2.67 fg	2.00 gh	2.00 gh	**2.20 e**
**Means**	**-**	**19.00 a**	**6.47 b**	**3.00 c**	**6.93 b**		**-**	**15.07 a**	**8.20 b**	**5.73 c**	**8.80 b**	
			**(65.94)**	**(84.21)**	**(63.52)**				**(47.58)**	**(61.97)**	**(41.60)**	
**LSD 5%**	**W = 0.67, C = 0.67, W×C = 1.50**						**W = 0.93, C = 0.93, W×C = 2.09**					

Means not sharing the same letter within a column differ significantly from each other at 5% probability level.

RETRACTED

Here, W = weed management strategies, C = wheat-based cropping systems, FW = fallow-wheat, RW = rice-wheat, CW = cotton-wheat, MW = mungbean-wheat and SW = sorghum-wheat, WF = weed-free, WC = weedy-check, FC = false seedbed, CC = herbicide application, AWE = allelopathic water extracts.

The RW cropping system observed the highest total weed density, whereas SW cropping system had the lowest total weed density during both years (Table 1). The interactive effect of WBCSs and WMSs had significant effect on total weed density (Table 1). All WBCSs with herbicide application recorded the lowest total weed density, whereas FW and RW cropping systems had the highest total weed density with weedy-check treatment during both years (Table 1).

### Density of broad and narrow-leaved weeds (m^-2^)

The WBCSs, WMSs and their interaction significantly altered the density of broad and narrow-leaved weeds. Weedy-check observed the highest density of broadleaved weeds, whereas weed-free treatment recorded the lowest density. Herbicide application resulted in the higher reduction in broadleaved weeds’ density than false seedbed and allelopathic water extracts during both year (Table 1). The FW and RW cropping systems observed the highest density of broadleaved weeds, whereas SW cropping system had the lowest density during both years (Table 1). Regarding interaction, the highest density of broadleaved weeds was noted in FW and RW cropping systems under weedy-check treatment, whereas the lowest density of broadleaved weeds was recorded for SW cropping system under all WMSs (Table 1).

Weedy-check treatment had the highest density of narrow leaved weeds, while herbicide application recorded their lowest density (Table 1). The RW cropping system noted the highest density, whereas SW cropping system observed the lowest density of narrow leaved weeds (Table 1). Regarding interaction, the highest density of narrow leaved weeds was observed in RW cropping system under weedy-check treatment, whereas SW cropping system under all weed management strategies observed their lowest density during both years (Table 1).

### Density of individual weeds (m^-2^)

Different WBCSs, WMSs and their interaction had significant effect on the density of individual weeds (Tables 2 and 3).

**Table 2:** Effect of different weed management strategies on density (m^-2^) of fat hen, common goosefoot, broad-leaved dock and yellow sweet clover under different wheat-based cropping systems during 2012–2013 and 2013–2014.

Cropping systems	2012–2013					Means	2013–2014					Means
	WF	WC	FS	CC	AWE		WF	WC	FS	CC	AWE	
	Fat hen											
**FW**	**-**	8.33 a	3.33 e	**-**	7.33 b	**3.80 a**	**-**	4.67 a	2.33 bc	**-**	1.67 cd	**1.73 a**
**RW**	**-**	6.33 c	3.67 e	**-**	5.33 d	**3.07 b**	**-**	2.67 b	1.33 d	**-**	1.33 d	**1.07 b**
**CW**	**-**	5.33 d	2.33 f	**-**	3.33 e	**2.20 c**	**-**	2.33 bc	1.33 d	**-**	1.00 d	**0.93 b**
**MW**	**-**	5.67 cd	2.33 f	**-**	3.67 e	**2.33 c**	**-**	2.67 b	1.33 d	**-**	1.67 cd	**1.13 b**
**SW**	**-**	3.33 e	1.33 g	**-**	1.67 fg	**1.27 d**	**-**	1.67 cd	1.33 d	**-**	1.67 cd	**0.93 b**
**Means**	**-**	**5.80 a**	**2.60 c**	**-**	**4.27 b**		**-**	**2.80 a**	**1.53 b**	**-**	**1.47 b**	
**LSD 5%**	W = 0.33, C = 0.33, W*C = 0.74						W = 0.16, C = 0.16, W*C = 0.32					
	**Common goosefoot**											
**FW**	**-**	20.33 a	8.00 h	**-**	14.33 d	**8.53 a**	**-**	9.00 a	5.00 d	**-**	5.33 cd	**3.87 a**
**RW**	**-**	17.33 b	9.33 fg	**-**	15.67 c	**8.47 a**	**-**	6.00 bc	4.00 e	**-**	5.33 cd	**3.07 b**
**CW**	**-**	16.00 c	8.33 gh	**-**	9.33 fg	**6.73 b**	**-**	6.67 b	2.33 gh	**-**	3.33 ef	**2.47 c**
**MW**	**-**	19.67 a	10.00 ef	**-**	11.00 e	**8.13 a**	**-**	5.67 cd	2.67 fg	**-**	4.00 e	**2.47 c**
**SW**	**-**	5.33 i	3.33 j	**-**	7.67 h	**3.27 c**	**-**	2.67 fg	1.33 i	**-**	1.67 hi	**1.13 d**
**Means**	**-**	**15.73 a**	**7.80 c**	**-**	**11.60 b**		**-**	**6.00 a**	**3.07 c**	**-**	**3.93 b**	
**LSD 5%**	**W = 0.48, C = 0.48, W×C = 1.07**						**W = 0.38, C = 0.38, W×C = 0.84**					
	**Broad-leaved dock**											
**FW**	**-**	131.00 a	23.00 h	**-**	58.33 e	**42.47a**	**-**	59.67 b	18.00 g	**-**	17.33 gh	**19.00 b**
**RW**	**-**	114.33 b	18.00 i	**-**	35.67 g	**33.60b**	**-**	110.67a	26.00 e	1.00 m	35.33 d	**34.60 a**
**CW**	**-**	76.33 d	8.00 jk	**-**	7.33 k	**18.33d**	**-**	21.33 f	9.00 ij	**-**	3.33 l	**6.73 d**
**MW**	**-**	98.33 c	17.67 i	**-**	25.00 h	**28.20c**	**-**	49.33 c	7.67 jk	**-**	10.67 i	**13.53 c**
**SW**	**-**	51.33 f	8.00 jk	**-**	11.33 j	**14.13e**	**-**	15.67 h	6.33 k	**-**	3.33 l	**5.07 e**
**Means**	**-**	**94.27 a**	**14.93 c**	**-**	**27.53 b**			**51.33 a**	**13.40 b**	**0.20 c**	**14.00 b**	
**LSD 5%**	**W = 1.58, C = 1.58, W×C = 3.52**						**W = 1.00, C = 1.00, W×C = 2.24**					
	**Yellow sweet clover**											
**FW**	**-**	4.33 b	1.67 fg	**-**	3.00 c-e	**1.80 b**	**-**	10.33b	5.33 d	**-**	1.67 g	**3.47 b**
**RW**	**-**	13.00 a	3.33 cd	**-**	3.67 bc	**4.00 a**	**-**	17.00 a	4.33 e	**-**	3.33 f	**4.93 a**
**CW**	**-**	3.33 cd	2.33 ef	**-**	2.67 de	**1.67bc**	**-**	7.33 c	2.33 g	**-**	2.00 g	**2.33 c**
**MW**	**-**	3.33 cd	2.33 ef	**-**	1.33 g	**1.40 c**	**-**	-	-	**-**	-	**-**
**SW**	**-**	2.33 ef	1.33 g	**-**	1.00 g	**0.93 d**	**-**	-	-	**-**	-	**-**
**Means**	**-**	**5.27 a**	**2.20 b**	**-**	**2.33 b**		**-**	**6.93 a**	**2.40 b**	**-**	**1.40 c**	
**LSD 5%**	**W = 0.36, C = 0.36, W×C = 0.81**						**W = 0.34, C = 0.34, W×C = 0.76**					

Means not sharing the same letter within a column differ significantly from each other at 5% probability level.

RETRACTED

Here, W = weed management strategies, C = wheat-based cropping systems, FW = fallow-wheat, RW = rice-wheat, CW = cotton-wheat, MW = mungbean-wheat and SW = sorghum-wheat, WF = weed-free, WC = weedy-check, FC = false seedbed, CC = herbicide application, AWE = allelopathic water extracts.

**Table 3:** Effect of different weed management strategies on density (m^-2^) of salt marsh and bermuda grass in various wheat-based cropping systems.

Cropping systems	2012–2013					Means	2013–2014						Means
	WF	WC	FS	CC	AWE		WF	WC		FS	CC	AWE	
	Salt marsh												
**FW**	-	7.67 cd	2.33 g-i	1.67 h-j	2.67 gh	**2.87 b**	**-**	4.33 d	2.33 fg		2.00 f-h	1.67 f-h	**2.07 b**
**RW**	-	21.00 a	6.67 de	2.33 g-i	8.33 c	**7.67 a**	**-**	14.33a	9.00 c		10.00 c	13.00 b	**9.27 a**
**CW**	-	6.33 e	1.67 h-j	1.00 jk	4.67 f	**2.73 b**	**-**	3.67 de	2.67 ef		1.33 gh	2.33 fg	**2.00 b**
**MW**	-	10.00 b	1.67 h-j	1.00 jk	3.33 g	**3.20 b**	**-**	4.33 d	1.67 f-h		1.00 hi	1.33 gh	**1.67 b**
**SW**	-	3.33 g	1.33 ij	0.67 jk	1.00 jk	**1.27 c**	**-**	2.67 ef	1.33 gh		1.00 hi	1.00 hi	**1.20 c**
**Means**	**-**	**9.67 a**	**2.73 c**	**1.33 d**	**4.00 b**		**-**	**5.87 a**	**3.40 c**		**3.07 c**	**3.87 b**	
**LSD 5%**	**W = 0.47, C = 0.47, W×C = 1.05**						**W = 0.46, C = 0.46, W×C = 1.03**						
	**Bermuda grass**												
**FW**	**-**	14.00 a	6.33 e	1.67 kl	2.67 ij	**4.93 a**	**-**	15.33 a	7.33 b		4.33 de	5.33 c	**6.47 a**
**RW**	**-**	12.00 b	5.00 f	2.00 j-l	4.33 fg	**4.67 a**	**-**	3.33 fg	1.33 h		1.00 h	1.33 h	**1.40 d**
**CW**	**-**	7.67 d	2.33 jk	2.00 j-l	1.67 kl	**2.73 c**	**-**	6.67 b	1.33 h		3.67 ef	7.33 b	**3.80 b**
**MW**	**-**	9.33 c	3.33 hi	1.33 l	2.00 j-l	**3.20 b**	**-**	5.00 cd	2.67 g		3.33 fg	1.33 h	**2.47 c**
**SW**	**-**	3.67 gh	1.67 kl	1.33 l	2.67 ij	**1.87 d**	**-**	1.67 h	1.33 h		1.00 h	1.00 h	**1.00 e**
**Means**	**-**	**9. 33 a**	**3.73 b**	**1.67 d**	**2.67 c**		**-**	**6.40 a**	**2.80 c**		**2.67 c**	**3.27 b**	
**LSD 5%**	**W = 0.41, C = 0.41, W×C = 0.92**							**W = 0.37, C = 0.37, W×C = 0.84**					

Means not sharing the same letter within a column differ significantly from each other at 5% probability level.

Here, W = weed management strategies, C = wheat-based cropping systems, FW = fallow-wheat, RW = rice-wheat, CW = cotton-wheat, MW = mungbean-wheat and SW = sorghum-wheat, WF = weed-free, WC = weedy-check, FC = false seedbed, CC = herbicide application, AWE = allelopathic water extracts.

Weedy-check treatment had the lowest density of fat hen, while herbicide application and weed-free treatments recorded its lowest density (Table 2). The FW cropping system had the highest density of fat hen, while SW cropping system resulted in its lowest density during both years (Table 2). Regarding interaction, the highest density of fat hen was noted for FW cropping system under weedy-check treatment, while all cropping systems with herbicide application had the lowest density of fat hen during both years (Table 2).

Weedy-cheek treatment recorded the highest density of common goosefoot, whereas herbicide application reduced its density nearly equal to weed-free treatment during both years (Table 2). The FW cropping system had the highest density of common goosefoot, whereas SW cropping system observed its lowest density (Table 2). Regarding interaction, the greatest density of common goosefoot was noticed in FW cropping system under weedy-check treatment and all cropping systems under herbicide application observed its lowest density (Table 2).

RETRACTED

Weedy-check treatment had the highest density of broad-leaved dock, while herbicide application decreased its density more than false seedbed and allelopathic extracts during both years (Table 2). The FW cropping system observed the highest density of broad-leaved dock in 2012–2013 and RW cropping system had its highest density in 2013–2014 (Table 2). However, SW cropping system observed the lowest density of broad-leaved dock during both years of study (Table 2). With respect to interaction, FW cropping system during 1^st^ year and RW cropping system during 2^nd^ year with weedy-check had the highest density of broad-leaved dock. All cropping systems under herbicide application had the lowest density of broad-leaved dock during both years (Table 2).

The highest density of yellow sweet clover was noted in weedy-check treatment, whereas herbicide application reduced its density almost similar to weed-free treatment during both years of study (Table 2). The RW cropping system noticed the highest density of yellow sweet clover, while SW cropping system observed its lowest density during both years (Table 2). Regarding interactive effect, RW cropping system with weedy-check treatment had the highest density of yellow sweet clover, whereas all cropping systems under herbicide application noted its lowest density during both years (Table 2).

The highest density of salt marsh was observed in weedy-check treatment, whereas herbicide application and weed-free treatments recorded its lowest density. The RW cropping system had the highest density of salt marsh, while SW cropping system noted its lowest density during both years (Table 3). The highest density of salt marsh was noticed in RW cropping system under weedy-check treatment, whereas its lowest density was noted in SW under all WMSs during both years (Table 3).

Weedy-check and weed-free treatments observed the highest and the lowest density of rabbit foot grass, respectively during each year (Table 3). The RW cropping system had the highest density of rabbit foot grass, whereas CW cropping system had no rabbit foot grass plant (Table 3). Regarding interaction, RW cropping system with weedy-check had the greatest density of rabbit foot grass, whereas CW cropping system under all WMSs had no rabbit foot grass plant during both years (Table 3).

Weedy-check observed the highest density of bermuda grass, while weed-free treatment had its lowest density (Table 3). The FW cropping system had the highest density of bermuda grass during both years (Table 3). However, SW cropping system had the lowest density of bermuda grass during both years (Table 3). Regarding interaction, the highest density of bermuda grass was observed in FW cropping system under weedy-check treatment, whereas its lowest density was noted in SW cropping system under all WMSs except few cases during both years (Table 3).

RETRACTED

## Discussion

Different WBCSs, WMSs and their interactions significantly altered weed diversity and density of total, individual, broad and narrow-leaved weeds. Weedy-check treatment recorded the highest densities and diversity, whereas weed-free treatment recorded lowest values in this regard. Different WMSs lowered diversity and density of weeds, and herbicide application proved better than all of the tested WMSs. Similarly, RW cropping system observed higher diversity and density of weeds, while SW cropping systems reduced density and diversity of weeds than rest of the WBCSs.

Herbicide application significantly decreased the density of weeds compared to weedy-check treatment [59]. However, excessive herbicide use is resulting in increases cases of herbicide-resistant weeds [37]. Therefore, integrated efforts are needed for successful weed management [38]. False seedbed can be used as an efficient strategy for integrated weed management [59, 60]. False seedbed managed weeds better than conventional seedbed [59, 61]. In the current study, false seedbed followed herbicide application in terms of density and diversity of weeds. Although, allelopathic extracts resulted in the lowest reduction in density and diversity, these are eco-friendly and successful against several weeds species. Sorghum allelochemicals are phytotoxic to growth of certain weeds such as *Chenopodium album*, *Phalaris minor*, *Avena fatua*, *Convolvulus arvensis* and *Rumex dentatus* etc. [47, 50, 62]. Sorghum roots exude an allelochemical “sorgoleone”, which negatively affects the performance of weeds [55, 63, 64]. Sunflower is another example of allelopathic crop and famous for its allelopathic chemicals such as sesquiterpene, lactones and terpenes [48, 65]. Brassica species also reduced seed germination of some species by releasing glucosinolates [66]. Therefore, mixture of sorghum, sunflower, ecuclptus, mulberry and brassica in alleopathic water extracts treatment helped in controlling density of weeds.

The RW cropping system increased weed diversity and density of total, broadleaved and narrow leaved weeds, while SW cropping system reduced these parameters (Tables 1–3). These findings are in contradiction with earlier work where FW and MW systems favoured grassy and broadleaved weeds, respectively [17]. The RW cropping system observed the highest density of yellow sweet clover, salt marsh, rabbit foot grass and corn spurry. Similarly, FW cropping system had the highest density of fat hen, common goosefoot, broadleaved dock and bermuda grass, while SW cropping system observed the lowest density of these weeds during both years (Tables 1–3). These results can be explained with the allelopathic potential of sorghum, which suppressed germination of these weeds. Several earlier studies have reported strong allelopathic impact of sorghum on seed germination and growth of different weed species [47, 50, 67]. Pervious work has also confirmed that fat hen was favoured by SW cropping system, and common goosefoot, broadleaved dock and salt marsh were favoured by RW cropping system. Nonetheless, broad-leaved dock, salt marsh, yellow sweet clover, rabbit foot grass, perennial sow thistle, corn spurry and bermuda grass were favoured by FW cropping system [17].

RETRACTED

The possible reason for weed suppression by SW cropping system is the crop sequence that created varying patterns of resource competition, allelopathic interference, soil disturbance and mechanical damage, which eventually resulted in unstable and frequently inhospitable environment for proliferation of weeds [68]. All variations that came due to cropping system affected weed seed bank. Fortunately, weed seed bank composition, density and diversity all are affected by cropping systems [69–72]. Higher weed density was noticed in RW cropping systems that may be due to less effect on weed seed bank.

The SW cropping system not only reduced weed density, but also limited weed flora. The suppression of weeds may be due to the allelopathic effects of sorghum in this cropping system. The similar idea was given by Liebman and Dyck [73] who proposed that crop rotation could be used as a weed management strategy as some crops in the rotations suppressed weeds by competing for resources and causing allelopathic disturbance. Many researches supported this idea and allelopathic nature of sorghum [51, 67, 74]. Sorghum possesses more allelopathic properties from root exudation and root and stem residual biomass [75]. Therefore, it can be used in reducing weeds in wheat, barley, corn, mungbean, *Brassica* and other crop species [76–79]. Weed reduction can range as high as 75% by sorghum as cover crops [79]. Allelochemicals from several crops has been identified and their activities for weed management have been reported [80]. Crops with powerful allelopathic potential are useful in weed management as sorghum residues could reduce weed population by 95% [81]. It secretes secondary chemical compounds that directly or in directly pose harmful or beneficial effects on plants [82]. Thus, SW cropping system adversely affected weed seed bank due to which this cropping system not only reduced weed density but also suppressed the weed flora.

RETRACTED

## Conclusions

The density and diversity of weeds was significantly altered by different weed management strategies, wheat-based cropping systems and their interaction. Although herbicide application performed better but it cannot be recommended because of its negative impacts on environment and ecosystems. Fortunately, allelopathic water extracts and false seedbed helped in managing weeds in eco-friendly way. The SW cropping system not only reduced weed density but also limited weed flora. It is concluded that false seedbed and sorghum-wheat cropping system can be used manage weeds in wheat-based cropping systems.
